# Prediction of the Age and Gender Based on Human Face Images Based on Deep Learning Algorithm

**DOI:** 10.1155/2022/1413597

**Published:** 2022-08-24

**Authors:** S. Haseena, S. Saroja, R. Madavan, Alagar Karthick, Bhaskar Pant, Melkamu Kifetew

**Affiliations:** ^1^Department of Information Technology, Mepco Schlenk Engineering College, Sivakasi, 626005 Tamil Nadu, India; ^2^Department of Electrical and Electronics Engineering, PSR Engineering College, Sivakasi, 626140 Tamil Nadu, India; ^3^Renewable Energy Lab, Department of Electrical and Electronics Engineering, KPR Institute of Engineering and Technology, Coimbatore, 641407 Tamil Nadu, India; ^4^Department of Computer Science and Engineering, Graphic Era Deemed to Be University, Bell Road, Clement Town, 248002 Dehradun, Uttarakhand, India; ^5^Department of Environmental Engineering, College of Biological and Chemical Engineering Addis Ababa Science and Technology University, Addis Ababa, Ethiopia

## Abstract

In recent times, nutrition recommendation system has gained increasing attention due to their need for healthy living. Current studies on the food domain deal with a recommendation system that focuses on independent users and their health problems but lack nutritional advice to individual users. The proposed system is developed to suggest nutritional food to people based on age and gender predicted from their face image. The designed methodology preprocesses the input image before performing feature extraction using the deep convolution neural network (DCNN) strategy. This network extracts *D*-dimensional characteristics from the source face image, followed by the feature selection strategy. The face's distinctive and identifiable traits are chosen utilizing a hybrid particle swarm optimization (HPSO) technique. Support vector machine (SVM) is used to classify a person's age and gender. The nutrition recommendation system relies on the age and gender classes. The proposed system is evaluated using classification rate, precision, and recall using Adience dataset and UTKface dataset, and real-world images exhibit excellent performance by achieving good prediction results and computation time.

## 1. Introduction

In recent years, many real-life applications such as social media, security control, advertising, and entertainment have made use of information contained in a human face. Automatic age [1] as well as gender [2] prediction from facial image plays a vital role in interpersonal communication and is always a significant area for researchers of computer vision [3]. Face age and gender recognition are a very important aspect of face analysis that has piqued the interest of researchers in areas such as demographic information collection, surveillance, human-computer interaction, marketing intelligence, and security. Recently nutrition recommendation has gained attention among both healthy and unhealthy people. This paper focuses on recommending nutritional advice for people based on their age and gender.

Different methodologies have been available to identify gender based on human biometric traits, mannerisms, and behaviours. A face provides distinguished information about a person that includes age, gender, expression, mood, ethnicity, etc. Gender identification from a person's face image is a difficult application in the computer vision community, image analysis, and artificial intelligence that recognises gender based on masculinity and femininity. It is binary classification problem which assigns a gender class to an individual. Gender identification is one part of facial analysis [4, 5] which focus on classifying the images under a controlled environment. There is a need for gender classification under an uncontrolled environment which is proposed in [6]. The gender of a person provides supplementary information that helps to retrieve fast and accurate information using human inspection whereas it is a challenging problem for computers.

Research efforts are taken to automatically predict the age from the face of a person [7]. The proposed method focuses by obtaining age-specific characteristics from face image, followed by age classification. The age of a human can be estimated using ageing cues present in the face image. Skin changes also help in perceiving the age of the adults. Age identification [8] is a complex process that depends on gender, race, ethnicity, lifestyle, make-up, and other external factors. Accurate facial age prediction remains challenging as the exact age differs from predicted age. Some public age recognition datasets include classifications such as child, teenager, adolescent, intermediate, and senior citizens.

The recommendation system suggests nutritional advice for the individual user based on their choice. In 2016, the World Health Organization [9] predicted that nearly 650 million people aged 18+ are overweight. Diet-related issues mainly, overweight and obesity are becoming the main reason for death throughout the world [10, 11]. A proper dietary plan is required to enhance people's standard of living. Therefore, a recommendation system for nutritional food consumption would be an appropriate solution for people with a busy lifestyle.

The planned nutrition recommendation system is depicted in Figure 1. This method captures a person's face as well as predicts their age and gender. Nutrition recommendation is provided to them based on this prediction.

The proposed system obtains the input from the dataset or through the real-time camera. Preprocessing is carried out to make it ready for further processing. DCNN is performed on the preprocessed image to retrieve the important features. Following that, feature selection is performed using hybrid particle swarm optimization (HPSO). The gender has 2 classes (male and female), and age of a person is classified into 8 age classes as “0–2,” “4–6,” “8–13,” “15–20,” “25–32,” “38–43,” “48–53,” and “60+” which is classified using support vector machine (SVM). The recommendation system provides nutritional advice based on the age and gender predicted for the individual. This main idea of the research are summarised below:

- A nutrition recommendation framework is developed to provide nutritional advice based on the user's age and gender
- DCNN is utilized for feature extraction, which learns relevant characteristics by retrieving distinctive features
- HPSO is used to select the best features in the image
- Combining DCNN with HPSO improves the computation time and accuracy
- SVM classifies age and gender
- The model is robust and surpasses the conventional scheme in contexts of classification rate, precision, and recall, as demonstrated by experiments on the Adience dataset and real pictures

The plan of the recommendation system is described in the following.  Section 2 articulates relevant research on age and gender. The conceptual methodology is detailed in Section 3.  Section 4 goes into detail about the exploratory designs, and Section 5 elaborates the performance evaluation.  Section 6 discusses the conclusion of the research.

## 2. Literature Survey

People's interest in nutrition recommendation systems has grown in recent years due to their relevance to healthy living. Existing nutrition recommendation systems suggests nutritional food for the people based on their health condition and individual preferences by getting input from the user. The proposed work automatically captures the face of a person and predicts their age and gender. Nutritional advice is recommended for a person based on their age category and their respective gender. Existing research works related to face are discussed in detail.

### 2.1. Face Detection and Identification

It is an important module of any face recognition system which should be more accurate and fast. Face detection algorithms are inspired mainly from object detection approaches. Region-based object detection classifies the generated object proposals. Each suggestion is classified as a face or nonface using a classifier. Hyperface [12] is a hierarchical multitask training architecture to conduct face identification, landmark mapping, posture prediction, and gender recognition. Region-based processing is faster. R-CNN [13] employs the region proposal network (RPN) [14], a tiny CNN. It predicts whether there is a sliding on the last feature map object or not and also predicts the boundary of those objects. RPN aids in the reduction of unnecessary face recommendations and the enhancement of their level. Face detection is generated at every place in a feature space at a particular scale using sliding window approaches. It is based on the feed-forward convolutional network. It has a shallow filter that can forecast object classifications and perform detection at multiple scales. Several facial tasks, such as facial attribute inference [15], face verification [16–19], and face recognition [20, 21], need the recognition and labeling of facial landmarks.

### 2.2. Gender Identification

Gender authentication may be done using a variety of data, including face photographs, hand skin photos, and physiological movements [22, 23], which contains a poll on gender detection systems utilizing face photos. Gender identification may be divided into two categories, according to [24, 25] (i) geometric oriented recognition and (ii) texture oriented recognition. Golomb et al. [26] proposed work on human gender detection that relies on neural networks. In gender detection, neural networks [27] were commonly employed for feature retrieval and categorization. Backpropagation neural networks are used in [28–30] for gender recognition. Furthermore, CNN has subsequently been found to be effective in obtaining exclusionary features and distinguishing genders [31, 32]. SVM, LDA, and AdaBoost are a few of the classification algorithms utilized in visual gender detection.

### 2.3. Age Identification

The person's face carries a great deal of information, including individuality, emotion, attitude, maturity level, ethnicity, race, and gender [33], which provided a detailed study of age modeling approaches using face photos. Kwon and Lobo [34] suggested a strategy for classifying photos into distinct age categories based on face characteristics by computing ratios of different metrics. This strategy, however, may not be appropriate for photographs with a lot of fluctuations in position, lighting, emotion, or blockage. The extraction of features is an important step in predicting human age. Active appearance model (AAM) [35], local binary patterns (LBP) [36–38], anthropometric features [39], and biologically inspired features (BIF) [40] are some of the feature extraction approaches that have been developed.

### 2.4. Deep Learning Methods

The initial deep learning technology utilized in a ML algorithm [41–43] was the deep neural network (DNN) [44, 45]. However, DNN has an overfitting problem and takes much too long to train. During learning, DNN was enhanced by utilizing limited Boltzmann machines (RBMs) and a deep belief network (DBN) [41, 46, 47]. DBN learning is quicker than DNN due to the inclusion of RBM. The RBMs are stacked DBM with unguided connections across the levels [48–53].

### 2.5. Feature-Based Methods

He et al. [54] proposed a linear appearance based method called principle component analysis (PCA). PCA is unsuitable for classifying because it maintains undesired intra-person differences when used for biometrics.

Babu et al. [55] proposed another linear appearance based method that classifies objects into sets of measurable object features called linear discriminant analysis (LDA). LDA has been more sensitive towards the training set's specific selection, resulting in lower outcomes than PCA.

To depict a diverse face expression, Donato [56] employed independent component analysis features using support vectors. Several researchers use it to analyse faces and facial expressions [57, 58]. Kernel PCA (KPCA) was proposed by Tanaka et al. [59], a nonparametric technique on the data to determine direction and minimize high dimensions.

Several nature-inspired techniques, such as PSO [60], GA [61], and ACO [62], have recently been employed for feature selection. In comparison to the previous techniques, GWO [63] is a novel methodology based on wolf chasing strategy. Wolf communities are created at random, which might lead to a lack of variation among wolves throughout the search process. This has a significant influence on the eventual solution's global convergence rate and efficiency. Thus, a novel approach is proposed to overcome this drawback.

### 2.6. Nutrition Recommendation System

Many works have been proposed for food recommendation which obtains the information from the user based on their preferences [64]. The collaborative filtering method [65] considers users' interest and makes predictions. But most of the systems do not suggest healthy and dietary food recommendations. Krizhevsky et al. proposed a dietary advice system [66] for individuals with diabetics. This system using k-means and SOM for clustering the food and suggests substitutes based on nutrition and food.

## 3. Proposed Work

The research work includes preprocessing, feature extraction, feature selection, age and gender categorization, and nutrition recommendation.  Figure 2 depicts the planned framework's block diagram, which is explored in depth below.

### 3.1. Image Preprocessing

It has a strong favourable impact on the quality of feature retrieval and the outcomes of image exploration. This is a combination comprising enhancements and enrichments that is required for a face recognition pipeline. Thus, image processing chores include noise subdual, contrast enrichments, and removal of undesirable effects on detention such as blurring by motion effects and color alterations.

#### 3.1.1. Noise Removal Using Mean Filter

Filtering is a technique for modifying and enriching an image. The main objective of such effects is to reduce noise, but they could be used to accentuate specific characteristics. 2D filtering techniques are typically considered an extension of 1D signal processing theory in image processing. The type of work, as well as the kind and characteristics of the data, frequently influences the filter selection. A mean filter is a basic linear filter that is both spontaneous and straightforward to use as a means of picture leveling. It aids in decreasing the degree of intensity fluctuation between pixels. It is commonly used to minimize picture noise. The primary principle behind mean filtering is to replace individual pixels value in a picture with the mean value of its neighbors, including itself. It has the potential to remove image pixels which are out of place in respective context. It is built round the kernel that represents the form and area of the neighborhood to be tested while computing the mean. A 3 × 3 square kernel is often employed, although a 5 × 5 square kernel could be utilized for extreme flattening. The two main difficulties with mean filtering are as follows:

- Singular pixel having an uncertain frequency that can have a negative impact on the total mean for other relevant pixels among its vicinity
- If there is an overlaps on the edge, the image becomes blurred

Two of the above concerns are handled using the median filter, that is, usually a superior noise-reduction filter over the mean filter though it takes longer to calculate.

#### 3.1.2. Face Detection and Alignment Using Landmark Localisation

Facial detection is the fundamental phase in any face recognition process. A face detection method assists in finding any face portion of an image. A face detection system must be resistant to changes in stance, lighting, emotion, scale, skin color, occlusions, disguises, make-up, and so on. The proposed method identifies the 68 landmark points in the face using the Dlib library.

Facial keypoints include the nasal tip, ear margins, mouths edges, eye contours, and so on. Certain face landmarks are required for face orientation that is required for facial registration. Face alignment utilizes the eye position and the center point in the face [67]. Based on these factors, the input photo is cropped and scaled, having the size of the image set to 110 × 110. Facial recognition and alignment are crucial aspects in biometrics, gender categorization, and age estimation.

### 3.2. Deep Convolutional Neural Network (DCNN)

DCNN is a deep neural network architecture which helps to extract the unique and distinguishing features from the preprocessed input. It helps in reducing the original dimension of the image and represents it in reduced form in a lesser space. Even after the reduced dimension, the features generated from the DCNN procedure yield the equivalent outcome as the source picture.

Studies prove that DCNN [68] excellently captures image features that have multilayer neural network architecture. DCNN [69] has a variety of uses in face recognition and is extremely sophisticated in learning the image's properties. Adopting DCNN in the proposed work to extract age [70] and gender [71] features in the face provides promising results.

The proposed age and gender recognition problem is solved using the designed DCNN architecture. This network has a six layer architecture that comprises of 5 convolution layers and 2 fully connected layers. DCNN has a deep learning network which performs feature extraction and classification task. The input image given to the proposed system is preprocessed and cropped to size 110 × 110 based on the landmarks detected. The input to the system is 5 × 112 × 112 owing the inclusion of zero padding to the matrices. There are 5 convolutional layers, each accompanied by ReLU, batch normalisation (BN), and max-pooling, as well as a dropout layer. After the fifth set of convolutional layers, the first fully connected layer appears, continued by ReLU, BN, dropout, and a subsequent fully connected layer. The network's second fully connected layer outputs 512 features. For the dropout layer, the dropout ratio is chosen as 0.5. The conv1 layer has a filter of size 7 × 7 and the stride of 4 × 4. All the max-pool layers have a filter of size 3 × 3 and the stride of 2 × 2. The conv2 layer has a 5 × 5-size filter, while the final convolution layer has a 3 × 3-size filter. The features are passed to the softmax function to normalise 512 features.  Figure 3 depicts a conceptual illustration of the proposed DCNN architecture.

Therefore, feature extraction employing DCNN retrieves the distinctive, exact, and informative characteristics found in an individual's facial picture, which aids in classification.

### 3.3. Particle Swarm Optimization (PSO)

PSO [72] is relatively a well-known optimization approach for finding optimal solution from a set of available alternatives. PSO is an optimization method inspired by the cooperative nature of a group of birds or swarm. Swarms have knowledge of predicting the distance of the food from their present location, while searching for food. PSO is composed of a collection of components. Every component is represented as a point, and it searches for an optimum. These components travel about the search space based on their individual best position as well as position of the swarm or nearby neighbors. In PSO, every solution is “swarm,” and the potential solutions are called as “particles.” Initially, the swarms have their position and velocity at a time (*t*) since the particles are moving. They change their positions by comparing their own best solution with the best solution of the neighbor. Each particle remembers the position, where it had its best solution. So far, this algorithm is used in artificial neural network training. In this method, PSO algorithm is incorporated to select the related features for the classification tasks. It also provides an iteratively better candidate solution or features.

Every particle is initialized with random position and velocity. The fitness value *f*(*x*) is calculated for the particles using equ (1).

(1) $$\begin{array}{c} f\left(x\right)=\overset{n}{\underset{i=0}{\sum }}x_{i}, \end{array}$$

where *x*_*i*_ is the particle and *n* is the number of particles. The fitness value is then contrasted against the optimum value of the particle on the previous fitness values which are named as personal best (pbest). Using the personal best, the global best (gbest) value is generated. It is continued until the stopping criteria. The pbest, gbest, and the old velocities are used in updating the velocity which is shown in

(2) $$\begin{array}{c} v_{i}\left(\text{t}+1\right)v_{i}\left(\text{t}\right)+\left(c_{1}\times \mathrm{rand}\left(\right)\times \left(p_{i}^{\text{best}}-p_{i}\left(\text{t}\right)\right)\right)+\left(c_{2}\times \mathrm{rand}\left(\right)\times \left(p_{g\text{b}est}-p_{i}\left(\text{t}\right)\right)\right), \end{array}$$

where *t* represents time, new velocity is given by *v*_*i*_ (*t* + 1), the weighting coefficients for are given by *c*_1_and*c*_2_, *p*_*i*_(t) is the particle position *p*^best^ is the optimum location of swarm, and *p*_*i*_^best^ is *i*^th^ optimum known location. rand() gives uniformly random variables. Equation (3) can be used to modify the particle's location.

(3) $$\begin{array}{c} p_{i}\left(t+1\right)=p_{i}\left(t\right)+v_{i}\left(t\right), \end{array}$$

where *p*_*i*_(*t* + 1) is the newly updated position, *p*_*i*_ is the recent position, and *v*_*i*_ is the recent velocity. The particles try to change their positions using factors like present position (*p*_*i*_), present velocity (*v*_*i*_), distance between present position (*p*_*i*_) and pbest (*p*_*i*_^*best*^), and the distance between present position (*p*_*i*_) and gbest (*p*_*gbest*_). The algorithm of PSO is given below.

The features present in the face image, which comes from the CNN framework, are considered as particles for training. The application of PSO throughout the training phase improves the solution vector's outcome and shortens the execution time. Premature convergence is the fundamental downside of PSO, which is mitigated by hybrid PSO.

### 3.4. Hybrid Particle Swarm Optimization (HPSO)

To simulate the particles, hybrid PSO is a unique feature selection approach that integrates PSO with the genetic algorithm (GA) [73, 74]. As PSO reaches the local optimum quickly, this local optimum cannot be avoided in the search space, and it reaches premature convergence at the earliest stage, and hence, this causes PSO to obtain local optimum region. To overcome this drawback, PSO is combined with GA. Combining GA and PSO is advantageous by sharing information among the particles which helps in computation steps. The hybrid PSO is proposed by performing a crossover operation on global best particles obtained from PSO. The problem dependent performance is one of the disadvantages of stochastic approaches. Thus, the different parameter settings are needed to exhibit high performance. The variations in the speed concerning inertia concluded that PSO is problem-dependent. Hence, this can be avoided with the help of hybrid PSO. The algorithm of the hybrid PSO is explained below.

Population is initialized, and fitness value is calculated for the population using equation (1). The fitness value is initialized to *p*_*i*_^best^ if the intended fitness value is greater than *p*_*i*_^best^. If not, *p*_*i*_^best^ is assigned to *p*_gbest_. The velocity is updated using equation (2), and the position is updated using equation (3). The crossover operation is added to the PSO algorithm to make it as a hybrid. The crossover is an operator in genetic algorithm preferably called recombination. Basically, there are various types of crossover used in genetic algorithm; here, single point crossover is used. In single point crossover, a random point is fixed, and the parent and the child are interchanged to produce the output of the crossover. The crossover is executed over the best solutions of PSO. The execution time is reduced with a hybrid PSO algorithm, used for training.

Hybrid PSO is carried out by the crossover operation of the best particles which are obtained from the PSO. The best particles are obtained by performing fitness calculations to each particle and compare these particles with others to get the pbest values or features. These personal best values are compared with other particles to acquire the global best particles. Later, these global best particles are given as input to crossover. Thus, the results are obtained, and the velocity and the positions are updated.

### 3.5. Age and Gender Classifications

Identity refers to the factors which differentiate one face from another. It can be age, gender, facial expression, and facial landmarks. The proposed system considers identity as the age and gender classifications. The proposed method uses classification to determine the age and gender of a human based on the input image. To categorize the age and gender, the classification procedure uses SVM [75].

SVM assists to understanding the attributes present in image and carry out the classification. SVM constructs an ideal hyperplane in multidimensional space, which aids in the categorization of images into two classes in gender categorization and eight classes in age categorization. The results of HPSO is mapped into the multidimensional space. The maximum marginal hyperplane (MMH) helps in distinguishing the classes.  Figure 4 shows the classification based on age and gender.

## 4. Experimental Results

The proposed system exhibits excellent performance by achieving a good classification of age and gender with reduced computation time and higher accuracy and also suggests nutritional advice for the user. The proposed system receives the input picture either by selecting it through the dataset or perhaps in real-time via the webcam. The source image is preprocessed to enhance the matching process's efficiency. The entry to the convolution network is 5 × 112 × 112 significantly with the addition of zero padding to the matrix of size 110 × 110. The landmark points present in the face are detected which helps to align and localize the face regions. The preprocessing procedures for the input facial image are depicted in Figures 5(a) input image, 5(b) face landmark, and 5(c) face detection.

The next phase in the proposed framework is feature extraction, which finds the characteristics that represent the face picture. The collected distinctive features from image will enhance the precision and performance of the system. These image characteristics are retrieved using DCNN and are distinct, allowing one class to be distinguished from another (for both age and gender). This network has a six-layer architecture that comprises of 5 convolution layers and 2 fully connected layers. These layers are then proceeded by a softmax layer at the last, which extracts 512 unique features.  Figure 6 depicts the features retrieved by DCNN as a consequence of the feature extraction method.

Once the features are extracted, feature selection is performed using HPSO which reduces the number of features extracted by DCNN. This helps in further reducing the image dimension and helps in improving the execution time.

Feature selection is then proceeded by the classification process which classifies the face image in terms of age and gender. Age is categorized into 8 classes as (0–2), (4–6), (8–12), (15–20), (25–32), (38–43), (48–53), and (60–100), and gender is categorized as male/female.  Figure 7 shows the result of classification.

Figure 8 depicts the classification output for men across all eight categories.  Figure 9 depicts the classification output for females across all eight categories.

Figure 10 illustrates the system's output for the provided source image, which displays the matching image as well as the relevant age and gender category.

The recommendation system suggests nutritional advice for the individual user based on their age and gender. Figure 10 depicts the system's recommendations based on predicted age and gender class.

## 5. Performance Evaluation

In this part, the recommended system's performance is compared and assessed against current methodologies. To assess the effectiveness of the current research, publicly available datasets like Adience and real-world images are used for experimentation purposes. Experiments are conducted in order to determine the age and gender of an input facial picture.

### 5.1. Implementation Details

Proposed system is implemented using Python TensorFlow framework. The input images are loaded using OpenCV while the dataset is split into train and test sets. Image preprocessing would be the first step that is performed on all images in the dataset to generate an image of size 112 × 112. Facial landmarks are detected and extracted using dlib and OpenCV. The location of 68 (*x*, *y*) coordinate points mapping to the structures on the face is estimated using the dlib library.  Figure 11 shows the 68 coordinate points detected in the input image using Dlib library. It then proceeds with alignment and localization of keypoints. Deep convolutional neural network (DCNN) is constructed and implemented in Python with the TensorFlow framework. The filter size starts from 32 and doubles in each convolutional layer until it reaches 512. Max pool layer is made up of 2 × 2 filters with a stride of 2. The dropout rate has been set at 0.5. To test the efficiency of the recommended system, publicly available datasets such as Adience and real-time photos are employed.

### 5.2. Dataset Description

The Adience dataset [76] is made up of photographs that were regularly published to Flickr by a smartphone. The Adience dataset, which comprises benchmarks of face pictures, is primarily utilized for age and gender recognition. The collection includes photographs with varying degrees of look, noise, stance, and lighting, as well as images obtained without rigorous planning or positioning. This dataset contains images of ages in 8 categories, namely, (0-2, 4-6, 8-13, 15-20, 25-32, 38-43, 48-53, 60+), and contains both the genders of images. The Adience face dataset is shown in Table 1, along with the face distribution across age categories and the total photos per category for men and women. Real-world images are also used which includes socially available face images and images that are captured in real time using a web camera.

### 5.3. Performance Metrics

The intended work's performance is measured in terms of classification rate, precision, and recall.

It is represented as

(4) $$\begin{array}{c} \text{Classification rate}=\frac{\text{No}.\text{of correctly classified Images}}{\text{ Total no}.\text{of images}}\times 100. \end{array}$$

Further, the precision and recall are calculated using

(5) $$\begin{array}{c} \text{Precision}=\frac{\text{ TP}}{\text{ TP}+\text{FP}}\times 100, \end{array}$$

(6) $$\begin{array}{c} \text{Recall}=\frac{\text{TP}}{\text{TP}+\text{FN}}\times 100, \end{array}$$

where TP represents the true positive, TN represents the true negative, FP represents the false positive, and FN represents the false negative.

### 5.4. Image Preprocessing

Importance of image preprocessing in the proposed system enhances the input image and prepares it for the next step in the recommendation system. The preprocessing step achieves improved accuracy, sensitivity, and specificity. Thus, using efficient preprocessing algorithms for image filtering, face detection, and face alignment makes the proposed system robust.  Figure 12 shows that there is an increase in the performance when the image preprocessing module is incorporated in the proposed system.

### 5.5. Feature Extraction

It is an essential step for automated methods which helps in extracting unique features from the given image. It helps in dimensionality reduction by mapping from a multidimensional space into a space of lesser dimensions. The proposed DCNN-based feature extraction technique is evaluated with other existing techniques such as SIFT [77], histogram of oriented gradients [78], LBP [79], and ICA [80]. The empirical findings of several feature extraction strategies are shown in Figure 13.

### 5.6. Feature Selection

Feature selection is also a dimensionality reduction method that helps in discarding irrelevant features by retaining only the discriminatory features. Several feature selection approaches such as GA, PSO, and ACO are evaluated with the proposed hybrid PSO-based feature selection strategy. The empirical findings of several feature selection strategies are shown in Figure 14.

### 5.7. Evaluation with State-of-the-Art Methods

The developed age and gender classification approach was evaluated using the Adience dataset and some real-world images. Simonyan and Zisserman [80] introduced the VGG network architecture which consists of a simple network with 3 × 3 convolutional layer stacked one above another. It consists of max pooling, two fully connected layers, and softmax classifier. The 16 and 19 in the VGG network represent the total number of hidden layers (weight layers). VGG network suffered from convergence and took huge time for training, and the architecture is very large. Szegedy et al. [81] introduced the inception network. This network extracts multilevel features with different convolutional layers of sizes 1 × 1, 3 × 3, and 5 × 5.

The proposed system is compared with VGG16, VGG19, and InceptionV3 models by statistical analysis using classification rate, precision, and recall.  Table 2 demonstrates that the developed method achieves superior result in classification, precision, and recall.

### 5.8. Execution Time

The execution time of various methods is compared.

#### 5.8.1. Measure of Execution Time with CNN Only

The CNN resulted in high execution time of 68 seconds approximately. This is because CNN used all the features that are retrieved. There is a comparatively large number of features that are obtained from CNN. Hence, due to numerous feature comparisons, the execution time on CNN is more than other methods. The execution time for CNN is approximately 68 seconds.

#### 5.8.2. Measure of Execution Time with CNN + PSO Method

This is varied method of selecting the best features using CNN + PSO. The features of the face images are reduced. It took lesser time than CNN since the face retrieval uses a lesser number of features which makes the execution faster. CNN-PSO takes 45 seconds approximately for face retrieval of the top 10 images.

#### 5.8.3. Measure of Execution Time with CNN + Hybrid PSO Method

The execution time is further reduced by CNN + hybrid PSO because of the crossover operation. The resulted execution time is approximately 4 seconds to classify the input image. The time is optimized as the features of the face images are optimized. The execution time for the three methods is depicted in Table 3.

### 5.9. Misclassifications

Misclassification rate also called as error rate defines the number of images wrongly classified in terms of age and gender. Some examples of age and gender misclassifications are provided in Figures 15(a) and 15(b), respectively. The results show that these misclassifications are due to the exceptionally varying conditions in the dataset as well as in the real-time image collected. Most of the misclassifications are caused because of occlusions in the face portion, low resolution/blur images, and side positions of the face. Gender misclassification occurs mainly for babies/kids and sometimes based on the hairstyle where the gender attributes are not completely differentiable. The misclassification rate is defined as

(7) $$\begin{array}{c} \text{Misclassification Rate}=\frac{\text{ FP}+\text{FP}}{\text{ TOTAL}}\times 100. \end{array}$$

The misclassification rate produced in the proposed system is 1.315%.

## 6. Conclusion and Future Work

For a wide range of applications, age and gender are critical factors. The scientific community has been more interested in estimating age and gender through facial photographs. This research offers a revolutionary nutrition recommendation system depending on age and gender detection from a facial image. Most of the existing nutrition recommendation system provides nutritional advice based on the information entered by the user manually or using the pathological reports. In this context, the current paper presents a recommender system which automatically captures the face and classifies the age and gender of an individual without any physical communication. Based on the classification results, nutritional recommendation is listed to the users. This paper incorporates DCNN, HPSO, and classification. Experiments reveal that the proposed system's age and gender recognition approaches exceed existing methods on the basis of accuracy and computational efficiency. In future, it is planned to develop group recommendation system for a group of users in public places.

## Figures and Tables

**Figure 1:** Overview of proposed nutrition recommendation system.

**Figure 2:** Proposed nutrition recommendation system.

**Figure 3:** Schematic diagram of the proposed network.

**Figure 4:** Classification of age and gender.

**Figure 5:** Image preprocessing: (a) input image; (b) face landmark; (c) face detection.

**Figure 6:** Features extracted from DCNN.

**Figure 7:** Classification results: (a) predicted age; (b) predicted gender; (c) combined output.

**Figure 8:** Classification results of males across all ages.

**Figure 9:** Classification results of females across all ages.

**Figure 10:** Nutrition recommendation based on predicted age and gender.

**Figure 11:** Visualization of 68 facial landmark coordinates in the dataset.

**Figure 12:** Performance of image preprocessing module for (a) age and (b) gender classifications.

**Figure 13:** Experimental results of feature extraction techniques.

**Figure 14:** Experimental results of feature selection techniques.

**Figure 15:** Misclassifications results of (a) age and (b) gender.

**Algorithm 1:** Algorithm for particle swarm optimization.

**Algorithm 2:** Algorithm of hybrid PSO.

**Table 1:** Adience dataset.

Gender	Labels in year								Total
	0-2	4-6	8-13	15-20	25-32	38-43	48-53	60+	
Female	682	1234	1360	919	2589	1056	433	427	9411
Male	745	928	934	734	2308	1294	392	442	8192
Both	1427	2162	2294	1653	4897	2350	825	869	19487

**Table 2:** Performance comparison of the proposed model with existing models.

Model	Classification rate (%)	Precision (%)	Recall (%)
VGG16	89.25	87.93	87.34
VGG19	90.71	89.48	90.83
Inception V3	93.61	93.78	92.86
Proposed age classification module	96.90	97.03	96.80
Proposed gender classification module	97.38	97.31	96.43
Proposed age and gender module	98.87	98.89	98.34

**Table 3:** Execution time of various methods.

Method	Execution time (in seconds)
Convolution neural network (CNN)	68 (approx.)
Convolution neural network with particle swarm optimization (CNN-PSO)	45 (approx.)
Convolution neural network with hybrid particle swarm optimization (CNN-hybrid PSO)	4 (approx.)

## Data Availability

The data used to support the findings of this study are included within the article.
